The article "Network Audio Data and Music Composition Teaching Based on Heterogeneous Cellular Network" was published in 2022. Journal: Comput Intell Neurosci.

# Network Audio Data and Music Composition Teaching Based on Heterogeneous Cellular Network

**DOI:** 10.1155/2022/9329856

**Published:** 2022-06-13

**Authors:** Qi Zhang

**Affiliations:** ^1^Art College, Shaoxing University, Shaoxing 312000, China; ^2^Faculty of Education, City University of Macau, Macau 999078, China

## Abstract

With the rapid development of services such as Industry 4.0 and Internet of Vehicles, it is difficult for traditional cellular networks to meet the needs of network users for quantification, diversification, and greenness in the future. Various cellular networks expand multiple micro-cell nodes and relay nodes under macro-cells to form a multilayer network architecture. Based on this, in the process of data transmission, the links have been repeatedly reduced, and at the same time, the terminal power consumption has been reduced and the running system has been improved. This article will use the ratio of the capacity, energy consumption, and resource allocation of different cellular networks as the main means to optimize the cost. Using graph theory, auction theory, and multipurpose optimization algorithms, we have conducted in-depth research topics on upstream and downstream wireless resource allocation, network relay deployment and transmission scheduling, MMW large-scale multi-antenna transmission technology, and base station energy management. A series of optimization schemes and algorithms are proposed. This dissertation is based on the research of educational system design theory in the field of educational technology so as to carry out the research of music education system design theory suitable for the nature of music subjects and learning and education characteristics. Based on the necessity and importance of music education system design theory, the research framework of music education system design theory is constructed in advance. The voice data acquisition system collects voice data through a network grabber and real-time recording and uses signal processing and pattern recognition technology to automatically classify the collected voice data into three categories: voice, environmental sound, and music. After establishing the audio data deployment strategy, simulation method, and architecture design based on heterogeneous cellular network, this paper designs the corresponding music composition teaching system, mainly including score editing, viewing, and content display of the composition teaching system, and the final test shows that the system designed in this paper can be effectively used in various music school teaching combined with heterogeneous cellular networks.

## 1. Introduction

With the rapid development of Internet technology, the number of user terminals and data traffic has increased dramatically, and the requirements for the performance and efficiency of future cellular communication systems have also increased. At the same time, the amount of mobile data in the world is also increasing rapidly, and Cisco predicts it will be 4 times. The annual average from 2017 to 2020 is more than 400 EB. Through the continuous advancement of mobile phone technology, data has gradually shown a lot of flowers and diversification, thus realizing the technological innovation and reform of cellular technology. Driven by this demand, Heterogeneous Cellular Networks (HetNets) composed of previous service stations and low-power nodes have appeared. The purpose is to improve the operating efficiency of the system's spectrum, continuously expand the capacity of the system, reduce the carrying capacity of the heat source station itself, and continuously increase the area covered by the indoor network, thereby further improving the quality of service (QoS). At the same time, the current planning of macro-base station sites is continuously deepening so that the distance between each other is constantly shrinking and presents a dense situation [1]. Coupled with the large-scale introduction of low-power nodes, the current environment of the cellular system will consume a large amount of energy, and as the use time increases, the problem becomes more prominent, and it also increases the difficulty of the network system operation, which brings problems to the optimization of the system [2].

Currently, in 5G dense heterogeneous cellular network, rational design of cellular architecture to make it play a better role is one of the key challenges. Adding many small cells to a macro-cell is one way to support the rapid growth of mobile data communications, provide high data rate services, and provide continuous coverage. However, a large number of network elements lead to a significant increase in power consumption. The optimization of network energy efficiency and the application of heterogeneous cellular networks in other fields have become research hotspots in academia.

In recent years, with the rapid development of the economic Internet, digital music platforms have become the focus of attention. Apparently, NetEase Cloud Music has a natural network gene, and it has close ties with different groups of people around the world. With the continuous improvement of NetEase's cloud computing technology, it uses a large amount of data provided by users to actively explore users' needs and preferences and continuously improve products. However, the educational status quo of music classroom education in the information age has not changed because of the development of information. At present, most schools still use the traditional music teaching mode.

This article introduces the technical theories related to the overall framework of the sound data acquisition system and uses the main technical theories including the following aspects, using the basic principles of Web cloning, advanced audio frequency transfer Linux sound architecture, and audio frequency data classification subsystem [3, 4]. Thus, the characteristics of VQT, decision tree and random forest classification algorithm models can be constructed. Finally, the PCA method is introduced in order to reduce the feature dimension, and the cross-validation principle is introduced to evaluate the performance of the classification model [5, 6]. The high cost of music hardware resources has always been the main reason for limiting music education resources. With the rapid development of computer technology and Internet technology, various music software are growing rapidly in front of the public. As a member, music education software adds new vitality to music education [7, 8]. These have their own characteristics. For those professionals with professional music literacy, they can carry out daily training of music scores in the music score database to provide them with music learning and training [9, 10]. There is also basic knowledge for ordinary people to learn music, and for others the focus is on music production and editing and music rhythm training.

## 2. Related Work

According to the literature, MIDI can be translated as “the digital interface of musical instruments.” This is the problem of electric audio musical instruments in the early 1980s in order to solve the communication problem [11, 12]. It is proposed in the literature that the energy efficiency measurement standards of cellular systems can be divided into three categories: component level, equipment level, and network level [13, 14]. The audio data acquisition system is mainly realized through Web crawler and real-time acquisition. It is proposed in the literature that real-time acquisition is mainly based on Advanced Linux Sound Architecture (ALSA). The literature regards the realization of the P2P mode as the main means to assist the education system [15, 16]. This method mainly takes into account the fact that streaming media technology is affected by bandwidth and cannot effectively transmit user information [17, 18]. Therefore, the P2P network docking technology is adopted to design and develop a network system based on the P2P architecture. The literature on decision tree algorithms is a type of statistics, data mining, and prediction methods that are widely used in the field of machine learning [19]. When the prediction target is a discrete value, the future target is continuously predicted.

StarC cloud integrated learning platform relies on the basic environment of StarC education cloud and integrates the construction of massive high-quality teaching resources, intelligent subject aids, online learning communities, and third-party services, and so on to promote the two-way integration of technology and education and realize the integration of education from the platform to the cloud application development. This time, the StarC comprehensive service cloud platform is used to integrate with this system, and the goal is to realize that the music education of many schools can be adapted to this system.

## 3. Audio Data Analysis Based on the Heterogeneous Cellular Network

### 3.1. Heterogeneous Cellular Network Deployment

#### 3.1.1. Heterogeneous Cellular Network Technology

In recent years, with the advancement of wireless communication technology, the birth and rapid development of the mobile Internet have been continuously advancing. Related to this, various handheld terminals such as smart phones and smart bracelets are growing rapidly. According to the latest data from Cisco, as of 2014, everyone in the world has a mobile terminal device. At the same time, smart terminals with powerful hardware computing capabilities, unique portable features, and rich smart applications (instant messaging, social networking, online games, video services, high-speed downloads, etc.) are slowly advancing. Personal desktop computers will replace mainstream user terminal devices and main data sources. Data services have undoubtedly increased the demand for broadband communications in cellular communication systems. For example, if the waiting time exceeds 100 milliseconds, the user will not be able to execute the online game application correctly [20].

Cellular mobile data has agglutination characteristics. In indoor scenarios, the quality of the channel between the macro-base station and indoor users is severely reduced due to the loss of the wall, so the method of ensuring indoor coverage is also a big problem [21].

The low-power nodes introduced in LTE-A mainly include the following four categories: Picocell, Femtocell, RelayNodes (RN), and RemoteRadioHead (RRH). This is shown in Table 1.

The low-power nodes introduced from LTE-A are mainly Picocell, Femtocell, RelayNodes (RN), and RemoteRadioHead. The transmission energy of Picocell is about 23 to 30 decibels, while the RemoteRadioHead is fixed at about 46 decibels. From the perspective of the corresponding radius, the radius of Picocell is wider, while the radius of RemoteRadioHead is only within 25 km.

#### 3.1.2. Deployment Strategy

In the same frequency network mode, when a user connects to a serving base station, its SINR is as follows:

(1) $$\begin{array}{c} \text{SINR}\left(x_{i}\right)=\frac{P_{i}h_{x_{i}}x_{i}^{-\alpha }}{I_{x_{i}}+\sigma^{2}}. \end{array}$$

*Base Station Power Consumption Model*. This chapter uses the power consumption model of the linear base station introduced in Chapter 1. In other words, the power consumption of a single macro-base station and a micro-base station is different.

(2) $$\begin{array}{c} P_{M,\text{tot}}=a_{M}\cdot N\cdot P_{M}+b_{M},\\ P_{m,\text{tot}}=a_{m}\cdot N\cdot P_{m}+b_{m}. \end{array}$$

Using probability geometry theory, the relationship between the average coverage performance of the system and the expansion parameters. This can guide the design of future development strategies. Although the same expressions are derived in the literature, they cannot be directly applied to the design of unfolding strategies, so in this chapter, please pay attention to whether they are suitable for transformation in order to draw more intuitive and interesting conclusions.

The user range probability is defined as follows:

(3) $$\begin{array}{c} P_{C}=\mathbb{P}\left[\text{SINR}>\gamma \right]. \end{array}$$

Based on the existing derived ideas and results in the literature, Theorems 1 and 2 are obtained through appropriate mathematical transformations as follows.

**Theorem 1 .**

In two different types of cellular networks composed of macro- and micro-base stations, the average range probability of users is as follows:

(4) $$\begin{array}{c} P_{C,SINR}\left(A\right)=\pi A\int_{t=0}^{\infty }\exp\left(-AC\left(\alpha \right)\gamma^{2/\alpha }t\right)\exp\left(-\gamma \sigma^{2}t^{\alpha /2}\right)\text{d}t. \end{array}$$

**Proof**

According to the definition of coverage probability in formula (3), we know that

(5) $$\begin{array}{c} P_{C,\text{SINR}}=\mathbb{P}\left(\underset{\varepsilon \left\{m,M\right\},x,\varepsilon_{i}}{\cup }\text{SINR}\left(x_{i}\right)>\gamma \right)=E\left[1\left(\underset{i\varepsilon \left\{m,M\right\},x,\varepsilon \phi_{i}}{\cup }\text{SINR}\left(x_{i}\right)>\gamma \right)\right]\overset{\left(a\right)}{=}\underset{i\in \left\{m,M\right\}}{\sum }E\underset{x,\varepsilon \phi_{i}}{\sum }\left[1\left(\underset{i\in K,x,\varepsilon_{†}}{\cup }\text{SINR}\left(x_{i}\right)>\gamma \right)\right]\overset{\left(b\right)}{=}\underset{i\in \left\{m,M\right\}}{\sum }\lambda_{i}\int_{{\mathbb{R}}^{2}}^{\overset{\left(c\right)}{=}}\mathbb{P}\left(\frac{P_{i}h_{x_{1}}l\left(x_{i}\right)}{I_{x_{i}}+\sigma^{2}}>\gamma \right)\text{d}x_{i}\underset{i\in \left\{m,M\right\}}{\sum }\lambda_{i}\int_{{\mathbb{R}}^{2}}{ℒ}_{I_{i}}\left(\frac{\gamma }{P_{i}l\left(x_{i}\right)}\right)e^{-r\sigma^{2}/p_{i}\left(x_{i}\right)}\text{d}x_{i}. \end{array}$$

Here, step (a) is obtained by “*γ*/>1 (0 dB), at most only one base station satisfies SINR *b* > *γ*.” Then,

(6) $$\begin{array}{c} {ℒ}_{I_{x_{j}}}\left(s\right)=\prod_{j\in \left\{m,M\right\}}E_{\phi ,\text{h}}\left[\prod_{x_{j}\in \phi_{j}/x_{i}}\exp\left(-sP_{j}h_{x_{j}}l\left(x_{j}\right)\right)\right]\\ =\prod_{j\in \left\{m,M\right\}}E_{\phi }\left[\prod_{{\text{x}}_{\text{I}}\in \phi_{j}/x_{i}}E_{\text{h}}\left[\exp\left(-sP_{j}h_{x_{j}}l\left(x_{j}\right)\right)\right]\right]\\ =\prod_{j\in \left\{m,M\right\}}E_{\phi }\left[\prod_{x_{j}\in \phi ,x_{i}}\frac{1}{1+sP_{j}l\left(x_{j}\right)}\right]\\ =\prod_{j\in \left\{m,M\right\}}\exp\left(-\lambda_{j}\int_{{\mathbb{R}}^{2}}\left(1-\frac{1}{1+sP_{j}x_{j}^{-\alpha }}\right)\text{d}x_{j}\right)\\ =\prod_{j\in \left\{m,M\right\}}\exp\left(-2\pi \lambda_{j}{\left(sP_{j}\right)}^{2/\alpha }\int_{0}^{\infty }r\int_{0}^{\infty }e^{\left(-t\left(1+r^{a}\right)\right)}dt\;dr\right)\\ =\exp\left(-s^{2/\alpha }C\left(\alpha \right)\underset{j\in \left\{m,M\right\}}{\sum }\lambda_{j}P_{j}^{2/\alpha }\right). \end{array}$$

Put equation (6) into equation (5) to get

(7) $$\begin{array}{c} P_{C,\text{SINR}}=\lambda_{M}\int_{0}^{\infty }2\pi r\text{exp}\left(-\left(\lambda_{M}P_{M}^{2/\alpha }+\lambda_{m}P_{m}^{2/\alpha }\right)C\left(\alpha \right){\left(\frac{\gamma }{P_{M}}\right)}^{2/\alpha }r^{2}\right)\\ \exp\left(-\left(\frac{\gamma }{P_{M}}\right)\sigma^{2}r^{\alpha }\right)\text{d}r+\lambda_{m}\int_{0}^{\infty }2\pi r\text{exp}\left(-\left(\lambda_{M}P_{M}^{2/\alpha }+\lambda_{m}P_{m}^{2/\alpha }\right)C\left(\alpha \right){\left(\frac{\gamma }{P_{m}}\right)}^{2/\alpha }r^{2}\right)\\ \text{exp}\left(-\left(\frac{\gamma }{P_{m}}\right)\sigma^{2}r^{\alpha }\right)\text{d}r. \end{array}$$

**Theorem 2 .**

If different types of cellular networks are used, the average coverage probability of users is as follows:

(8) $$\begin{array}{c} P_{C,RP}\left(A\right)=\pi A\int_{t=0}^{\infty }\text{exp}\left(-\pi A\left(1+Z\left(\gamma ,\alpha ,1\right)\right)t\right)\text{exp}\left(-\gamma \sigma^{2}t^{\alpha /2}\right)\text{d}t. \end{array}$$

Therefore, the range probability of the user can be expressed as follows:

(9) $$\begin{array}{c} A_{\text{k}}=\frac{\lambda_{k}P_{k}^{2/\alpha }}{\sum_{j\in \left\{m,M\right\}}\lambda_{j}P_{j}^{2/\alpha }},\\ O_{\text{k}}=\frac{2\pi \lambda_{k}}{A_{k}}\overset{\infty }{\underset{0}{\int }}\text{xexp}\left\{-\frac{\gamma \sigma^{2}}{P_{k}r^{-\alpha }}-\pi \underset{j\in \left\{m,M\right\}}{\sum }\lambda_{j}{\left(\frac{P_{j}}{P_{k}}\right)}^{2/\alpha }\left[1+Z\left(\gamma ,\alpha ,1\right)\right]r^{2}\right\}\text{d}r. \end{array}$$

Therefore, you can get

(10) $$\begin{array}{c} P_{C,RP}=\lambda_{M}\int_{0}^{\infty }2\pi r\text{exp}\left(\begin{array}{c} -\pi \left(\lambda_{M}+\lambda_{m}{\left(\frac{P_{m}}{P_{M}}\right)}^{2/\alpha }\right)\\ \left(1+Z\left(\gamma ,\alpha ,1\right)\right)r^{2} \end{array}\right)\text{exp}\left(-\left(\frac{\gamma }{P_{M}}\right)\sigma^{2}r^{\alpha }\right)\text{d}r\\ +\lambda_{m}\int_{0}^{\infty }2\pi r\text{exp}\left(\begin{array}{c} -\pi \left(\lambda_{M}{\left(\frac{P_{M}}{P_{m}}\right)}^{2/\alpha }+\lambda_{m}\right)\\ \left(1+Z\left(\gamma ,\alpha ,1\right)\right)r^{2} \end{array}\right)\text{exp}\left(-\left(\frac{\gamma }{P_{m}}\right)\sigma^{2}r^{\alpha }\right)\text{d}r. \end{array}$$

**Theorem 3 .**

In two different types of cellular networks composed of macro-base stations and micro-base stations, “*P*_*C*,SINR_(*A*)” and “*P*_*C*.*RP*_(*A*)” are the monotonic energy-dependent expansion coefficient *a* Increase the function. *A*_1_ and *A*_2_ are two positive numbers and satisfy *A*_2_ > *A*_1_ at the same time. Then,

(11) $$\begin{array}{c} P_{C,\text{SINR}}\left(A_{2}\right)=\pi A_{2}\int_{t_{2}=0}^{\infty }\text{exp}\left(-A_{2}C\left(\alpha \right)\gamma^{2/\alpha }t_{2}\right)\exp\left(-\gamma \sigma^{2}t_{2}^{\alpha /2}\right)\text{d}t_{2}\\ \overset{\left(a\right)}{=\pi A_{2}}\frac{A_{1}}{A_{2}}\int_{t_{1}=0}^{\infty }\text{exp}\left(-A_{2}C\left(\alpha \right)\gamma^{2/\alpha }\frac{t_{1}A_{1}}{A_{2}}\right)\text{exp}\left(-\gamma \sigma^{2}{\left(\frac{t_{1}A_{1}}{A_{2}}\right)}^{\alpha /2}\right)\text{d}t_{1}\\ =\pi A_{1}\int_{t_{1}=0}^{\infty }\text{exp}\left(-A_{1}C\left(\alpha \right)\gamma^{2/\alpha }t_{1}\right)\text{exp}\left(-\gamma \sigma^{2}t_{1}^{\alpha /2}{\left(\frac{A_{1}}{A_{2}}\right)}^{\alpha /2}\right)\text{d}t_{1}\\ >\overset{\left(b\right)}{\pi A_{2}}\int_{t_{1}=0}^{\infty }\text{exp}\left(-A_{1}C\left(\alpha \right)\gamma^{2/\alpha }t_{1}\right)\text{exp}\left(-\gamma \sigma^{2}t_{1}^{\alpha /2}\right)\text{d}t_{1}=P_{C,SNR}\left(A_{1}\right). \end{array}$$

**Theorem 4 .**

In two different types of cellular networks composed of macro-base stations and micro-base stations, if the expansion coefficient that depends on energy is applied, the average range probability of the system will be satisfied.

(12) $$\begin{array}{c} \frac{\pi \text{exp}\left(-\gamma \sigma^{2}T^{\alpha /2}\right)}{C\left(\alpha \right)\gamma^{2/\alpha }}\leq \underset{A⟶\infty }{\lim}P_{C,SINR}\left(A\right)\leq \frac{\pi }{C\left(\alpha \right)\gamma^{2/\alpha }},\\ \frac{\pi \;\exp\left(-\gamma \sigma^{2}T^{\alpha /2}\right)}{1+Z\left(\gamma ,\alpha ,1\right)}\leq \underset{A⟶\infty }{\lim}P_{C,RP}\left(A\right)\leq \frac{\pi }{1+Z\left(\gamma ,\alpha ,1\right)}. \end{array}$$

From (4), we can get

(13) $$\begin{array}{c} P_{C,\text{SINR}}\left(A\right)=\pi \int_{0}^{\infty }\text{exp}\left(-C\left(\alpha \right)\gamma^{2/\alpha }t\right)\text{exp}\left(-{\gamma \sigma }^{2}{\left(\frac{\text{t}}{A}\right)}^{\alpha /2}\right)\text{d}t\\ =\pi \int_{0}^{TA}\text{exp}\left(-C\left(\alpha \right)\gamma^{2/\alpha }t\right)\text{exp}\left(-\gamma \sigma^{2}{\left(\frac{t}{A}\right)}^{\alpha /2}\right)\text{d}t\\ +\pi \int_{TA}^{\infty }\exp\left(-C\left(\alpha \right)\gamma^{2/\alpha }t\right)\exp\left(-{\gamma \sigma }^{2}{\left(\frac{t}{A}\right)}^{\alpha /2}\right)\text{d}t. \end{array}$$

So when *A* ⟶ ∞, it converges to 0; we have

(14) $$\begin{array}{c} \underset{A⟶\infty }{\lim}\pi \int_{0}^{TA}\exp\left(-C\left(\alpha \right)\gamma^{2/\alpha }t\right)\exp\left(-\gamma \sigma^{2}{\left(\frac{t}{A}\right)}^{\alpha /2}\right)\text{d}t\\ =\underset{A⟶\infty }{\lim}\pi \int_{0}^{\infty }\exp\left(-C\left(\alpha \right)\gamma^{2/\alpha }t\right)\exp\left(-\gamma \sigma^{2}{\left(\frac{t}{A}\right)}^{\alpha /2}\right)\text{d}t\\ \in \left[\frac{\pi \;\exp\left(-\gamma \sigma T^{\alpha /2}\right)}{C\left(\alpha \right)\gamma^{2/\alpha }},\frac{\pi }{C\left(\alpha \right)\gamma^{2/\alpha }}\right]. \end{array}$$

Several indicators of networked energy efficiency are listed. This chapter uses Area Power Consumption (APC) to measure the energy efficiency of the system. Therefore, our problem can be expressed mathematically as follows:

*P*1:
  (15) $$\begin{array}{c} \underset{\lambda_{M}P_{M},\lambda_{m},P_{m}}{\text{minimize}}APC\\ \text{subjectto}P_{C}\left(\lambda_{M},P_{M},\lambda_{m},P_{m}\right)\geq P_{\exp}\\ P_{M,\max}\geq P_{M}\geq 0\\ P_{m,\max}\geq P_{m}\geq 0\\ \lambda_{M,\max}\geq \lambda_{M}\geq 0\\ \lambda_{m,\max}\geq \lambda_{m}\geq 0. \end{array}$$

The first constraint is that the average-range probability of the system is greater than the expected value. APC can be expressed as follows:

(16) $$\begin{array}{c} \text{APC}=\lambda_{M}\left(a_{M}NP_{M}+b_{M}\right)+\lambda_{m}\left(a_{m}NP_{m}+b_{m}\right). \end{array}$$

**Theorem 5 .**

If there is an optimal solution to problem *P*1, the optimal solution must satisfy the following equation:

(17) $$\begin{array}{c} \lambda_{m}P_{m}^{2/\alpha }+\lambda_{M}P_{M}^{2/\alpha }=A^{*}. \end{array}$$

Here, if you select the access mode according to the cell, you can use the following formulas to solve the problem:

(18) $$\begin{array}{c} P_{C,RP}\left(A^{*}\right)=P_{\exp},\\ P_{C,SNR}\left(A^{*}\right)=P_{\exp}. \end{array}$$

In a homogeneous cellular network, *λ*_*m*_ = 0, *P*_m_ = 0, *P*1 is as follows:

*P*2:

(19) $$\begin{array}{c} \underset{\lambda_{M},P_{M}}{\text{minimize}}\lambda_{M}\left(a_{M}NP_{M}+b_{M}\right)\\ \text{subjectto}\lambda_{M}P_{M}^{2/\alpha }=A^{*}\\ P_{M,\max}\geq P_{M}\geq 0\\ \lambda_{M,\max}\geq \lambda_{M}\geq 0. \end{array}$$

The above two-variable optimization problem can be simplified to a single-variable optimization problem by using equation constraints, and the optimal solution (optimal expansion strategy) can be obtained through the final solution:

(20) $$\begin{array}{c} P_{M}^{*}=\min\left(\max\left(\frac{2b_{M}}{a_{M}N\left(\alpha -2\right)},{\left(\frac{A^{*}}{\lambda_{M,\max}}\right)}^{\alpha /2}\right),P_{M,\max}\right),\\ \lambda_{M}^{*}=A^{*}P_{M}^{*-2/\alpha }. \end{array}$$

Using Theorem 5 in *λ*_*m*_=*P*_*m*_^−2/*α*^(*A*^*∗*^ − *λ*_*M*_*P*_*M*_^2/*α*^) to eliminate the variable *λ*_m_, we can get

(21) $$\begin{array}{c} APC=\lambda_{M}\left(a_{M}NP_{M}+b_{M}\right)+\lambda_{m}\left(a_{m}NP_{m}+b_{m}\right)=\lambda_{M}\left(a_{M}NP_{M}+b_{M}\right)\\ -P_{m}^{-2/\alpha }\lambda_{M}\left(a_{m}NP_{m}+b_{m}\right)P_{M}^{2/\alpha }+P_{m}^{-2/\alpha }A^{*}\left(a_{m}NP_{m}+b_{m}\right). \end{array}$$

Therefore, problem *P*1 is simplified to the following:

*P*3:

(22) $$\begin{array}{c} \underset{\lambda_{M},P_{M}}{\text{minimize}}\lambda_{M}G\left(P_{M}\right)\\ \text{subjectto}A^{*}\geq \lambda_{M}P_{M}^{2/\alpha }\geq A^{*}-\lambda_{m,\text{mar}}P_{m}^{2/\alpha }\\ P_{M,\max}\geq P_{M}\geq 0\\ \lambda_{M,\max}\geq \lambda_{M}\geq 0. \end{array}$$

Among them,

(23) $$\begin{array}{c} G\left(x\right)=a_{1}x-a_{2}x^{2/\alpha }\\ a_{1}=a_{M}N,a_{2}=P_{m}^{-2/\alpha }\left(a_{m}NP_{m}+b_{m}\right)+b_{M}. \end{array}$$

Problem *P*3 also has two variables, so it is difficult to solve the problem. For this purpose, we tried to simplify the problem further. Through observation and analysis of problem *P*3, the following conclusions can be drawn:

(24) $$\begin{array}{c} \lambda_{M}^{*}=\left\{\begin{array}{c} \text{max}\left(\frac{A^{*}-\lambda_{m,\max}P_{m}^{2/\alpha }}{P_{M}^{2/\alpha }},0\right)G\left({\text{P}}_{\text{M}}\right)\geq 0,\\ \text{min}\left(\frac{A^{*}}{P_{M}^{2/\alpha }},\lambda_{M,\max}\right),G\left({\text{P}}_{\text{M}}\right)<0. \end{array}\right) \end{array}$$

Bringing it into *G*(*P*_*M*_) ≥ 0, *A*^*∗*^ − *λ*_*m*,max_*P*_*m*_^2/*α*^ ≤ 0, the following univariate optimization problem can be obtained:

*P*4:

(25) $$\begin{array}{c} \underset{P_{M}}{\text{minimize}}0\\ \text{subjectto}P_{M,\max}\geq P_{M}\geq 0,\\ G\left(P_{M}\right)\geq 0. \end{array}$$

Bringing it into (*P*_*M*_) ≥ 0, *A*^*∗*^ − *λ*_*m*,max_*P*_*m*_^2/*α*^ > 0, the following univariate optimization problem can be obtained:

*P*5:

(26) $$\begin{array}{c} \underset{P_{M}}{\text{minimize}}\frac{A^{*}-\lambda_{m,\max}P_{m}^{2/\alpha }}{P_{M}^{2/\alpha }}\\ G\left(P_{M}\right)\text{subjectto}P_{M,\max}\geq P_{M}\geq 0\\ \lambda_{M,\max}\geq \frac{A^{*}-\lambda_{m,\max}P_{m}^{2/\alpha }}{P_{M}^{2/\alpha }}\geq 0\\ G\left(P_{M}\right)\geq 0. \end{array}$$

Bringing it into *G*(*P*_*M*_) < 0, *A*/*P*_*M*_^2/*α*^ ≤ *λ*_*M*,max_, the following univariate optimization problem can be obtained:

*P*6:

(27) $$\begin{array}{c} \underset{P_{3}}{\text{minimize}}\frac{A^{*}}{P_{M}^{2/\alpha }}G\left(P_{M}\right)\\ \text{subjectto}P_{M,\max}\geq P_{M}\geq 0\\ \frac{A^{*}}{P_{M}^{2/\alpha }}\leq \lambda_{M,\max}\\ G\left(P_{M}\right)<0. \end{array}$$

Bringing it into problem *P*3 and then considering the constraint *G* (*P*_*M*) < 0, *A*/(*P*_*M*^(2/*α*)) > *λ* (*M*, max), the following univariate optimization problem can be obtained:

*P*7:

(28) $$\begin{array}{c} \underset{P_{M}}{\text{minimize}}\lambda_{M,\max}G\left(P_{M}\right)\\ \text{subjectto}P_{M,\max}\geq P_{M}\geq 0\\ \frac{A^{*}}{P_{M}^{2/\alpha }}>\lambda_{M,\max}\lambda_{M,\max}\\ P_{M}^{2/\alpha }\geq A^{*}-\lambda_{m,\max}P_{m}^{2/\alpha }G\\ \left(P_{M}\right)<0. \end{array}$$

The above four cases are all univariate optimization problems. This function has good monotonic properties and can convert related constraints into linear constraints. As a result, problems *P*4 to *P*7 can be quickly solved. After discussing and solving the above four situations, the best solution to problem *P*3 can be obtained:

(29) $$\begin{array}{c} \left[\lambda_{M}^{*},P_{M}^{*},\lambda_{m}^{*}\right]=\left[\lambda_{M,i}^{*},P_{M,i}^{*},\lambda_{m,i}^{*}\right]. \end{array}$$

#### 3.1.3. Simulation Method

First, investigate the impact of energy saving threshold *Z* on system performance. The sleep strategy of the micro-base station introduced in this chapter is to investigate whether the performance of energy efficiency can improve the performance and to provide a reference plan for its research. The sleep strategy of micro-base stations has not been adopted. In other words, all micro-base stations are active, and this scheme is marked as REF. Corresponding to this, the sleep strategy of the micro-base station in this chapter is shown as ES.  Figure 1 shows the theoretical derivation solution (numerical solution of Monte Carlo simulation) and system-level simulation results under various user densities and various energy-saving thresholds. The channel noise power is set to *σ*^2^=−90 dBm.

The Monte Carlo simulation mainly uses random numbers to simulate images and outputs the approximate results of the research itself through the simulation input of a large number of samples. This time, a variety of different random numbers are used to realize the Monte Carlo simulation, which finally makes the results closer to the real needs.

In order to overcome this difficulty, a relatively simple method is to use 0, 1, and other energy saving limits. Therefore, it is possible to avoid a serious loss in complex calculations and spectral efficiency performance, as well as a reduction in ECR performance in an actual system.

#### 3.1.4. Architecture Design

Dr. Fang proposed a new cross-lingual wireless network architecture, namely, CCH (Cognitive Capacity Harvesting Networks) architecture. In this chapter, the above framework is applicable to different cellular network systems composed of macro-base stations and relays. It is defined as a multihop cellular network. In multihop, we propose 4 identifiable cellular network entities. SSP has its own cellular communication band (BasicBand). In addition, it can also detect a part of the noncellular frequency band that is idle for other networks (referred to as the relative primary network) so that Sketchup can provide better services. U can be a traditional device with an existing access technology, or a new device with a sensing function. In order to provide services to all SVs, SSP has developed multiple relay nodes and base stations capable of identifying SVs. These relay nodes and base stations form the basis of a cellular network and can work in BasicBand or HarvestedBand. If the SU has been identified, the relay node or base station can be accessed through BasicBand and HarvestedBand.

### 3.2. Audio Data Collection and Application

This article describes the main process of extracting new functions from the audio data classification subsystem and the training decision tree model and analyzes the fitting performance of the system classification model in the training data set. In order to completely test the resolution of the new features of surrounding sounds and music and the generalization ability of the decision tree model, this article uses a test data set completely different from the training data set to test the system. The test data contains approximately 8.4 hours of external audio and 14.6 hours of music audio. The test results are shown in Table 2.

From Table 2, it can be seen that the ratios of dimension feature + decision tree decision and sigma judgment are very high, most of which exceed 70%. Only the ratio of sigma judgment corresponding to the recall rate of ambient sound is relatively low.

In the system implementation process, the random forest of 50 trees and the error rate outside each bag are shown in Figures 1 and 2.

It can be seen from Figure 1 that as the number of trees increases, the error rate of each outsourcing shows a downward trend. When the number of trees is 5, the error rate of outsourcing classification decreases the highest and then gradually becomes smooth. When the number is 15, gradually tending to a low-speed decline, the subsequent outsourcing classification error rate is between 0.05 and 0.1.

Figure 2 is similar to Figure 1. As the number of trees increases, the outsourcing classification error first declines rapidly and begins to decline slowly when it decreases to 0.05, and the volatility thereafter is not large.

The number of training random forest trees is confirmed by the training method. Therefore, the number of trees used in the abscissa of this simulation is 50.

In addition to using the out-of-bag error rate to evaluate the performance of the random forest model for classification, the average cumulative classification margin can also be used to evaluate the model. The classification margin refers to the value of the maximum score difference of the observed sample. When it is wrongly judged as another category, the judgment is made based on the value of subtracting the maximum score from the decision tree.

In order to fully test the classification performance of the random forest model, this paper also uses the TUT data set to test the random forest model trained in this section. The specific test results are shown in Table 3.

## 4. Music Composition Teaching System Design and Practical Application

### 4.1. System Module Design and Implementation

The main function of the music editing module is to provide teachers with a real-time classroom music editing environment. The design features are as follows:

1. Special customized music scores taught in the classroom: The score editing module supports music notation, key notation, beat notation, performance speed, track number, playing instrument, and many other notation settings. Teachers can edit the necessary music scores based on the classroom instruction content that was difficult to achieve in music education in the past [22].
2. Editing music is convenient and fast. After the initialization, the scores are presented in the form of staff, and the teacher must fill the staff according to his educational needs [23]. Because the entire music editing module supports mouse and touch control operations, teachers can easily edit music according to their own teaching habits and actual classroom teaching situations.

#### 4.1.1. Design and Implementation of the Initialization Submodule for Music Score Editing

The new score contains records of score information such as part symbols, key marks, beat marks, track numbers, performance speed, and instrument types. The score editing module is mainly realized by WPF technology [24].

The new score is in two parts. The first part is to set the basic information of the score, such as the name of the score, the description of the score, the author, and copyright information [25]. The second part is the staff setting. This provides a general choice, such as tempo, playing speed, number of tracks, clef, key notation, playing instrument, and so on. Optimize data access technology so that users can use optimization technology to minimize the flow of access to necessary information [26]. The system cannot extract too complex related data to reduce the load on the server [27].

#### 4.1.2. Design and Implementation of the Score Editing Submodule

The main function of the music editing submodule is to edit music. It mainly includes the modification of notation, pitch mark, and beat mark: adding notes, points, and bars. Delete notes, dots, and so on in the notation method. The music editing submodule is the core submodule of the music editing module that contains complex and diverse music rules [28]. Its realization determines the accuracy and stability of music editing [29]. In order to improve the rendering effect, this module uses WPF technology. Through a detailed investigation of music teaching materials, the management status of music score editing is mainly analyzed from the point of view of music online education, which hinders the understanding of the music score editing process [30]. Regardless of whether the interaction of online data is realized, the education and learning of online data has been completed. There is close contact between the educational process and management functions.

#### 4.1.3. Design and Implementation of the Music Score Preview and Save Submodule

The main function of the submodule of score preview and save is to find problems and correct them within time. In this way, the guidance of music teachers in the classroom becomes much easier. The submodule interface adopts WPF technology, and the music performance and music storage module adopts MIDI technology. At the same time, in order to achieve an excellent presentation effect, the system uses the current mainstream VST software audio source technology to process. In the operation of high-performance music score database, it is not enough to focus on designing the best library table structure to make the best index. Optimizing queries, optimizing indexes, and optimizing the table structure of the score database must be closely related.

### 4.2. Design and Implementation of the Demonstration Module

The main function of the music presentation module is to combine audio images, play music at the same time, and link to display music. The design features are as follows:

1. *Joint Demonstration of Piano and Music*. Not only can it visually confirm the current performance position of the score, but also clearly confirm the performance method of the current position, which promotes students' music learning.
2. *Rich Interface Control*. In order to facilitate the teacher's demonstration in the classroom, a rich music interface control module has been added. For example, the teacher can use the zoom button to adjust the size of the music program, or use the button to display the piano to enlarge the score of the display area. In courses such as real-time performance, in order to easily switch the position of the piano and music, move up and down.
3. *Rich Performance Effects*. Change the key signs of the score presentation, select a specific score, and so on, and then cycle through the part of the presentation score. Through these multidimensional effects, students can more clearly understand the overall structure and audio-visual effects of the score.
4. *Good playback Sound Quality*. Improve the sound quality of the demonstration module so that teachers and students have a better sense of effect during use.

#### 4.2.1. The Design and Realization of the Score Playing Control Submodule

The main function of the music playback control submodule is to control the playback effects, such as selecting the playback track, selecting the playback sound, and selecting the playing instrument of each music track.

#### 4.2.2. Design and Implementation of the Score Display Control Submodule

In order to make it easier for teachers and students to use, various display effects are set, and the demonstration effects are more intuitive. This module is mainly implemented by WPF technology.

#### 4.2.3. Design and Realization of the Submodule of Music Score and Sound Effect Processing

The main function of the music sound processing submodule is to improve the effect sound of the score. In this case, the performance of music will become more professional and comfortable. This module is one of the important modules of music presentation, and it is also the most difficult place to implement. After a comprehensive study of all factors, we decided to use the current mainstream open source software audio source VST plug-in to improve the sound of music.

### 4.3. Test of the Music Composition Teaching System

With the continuous improvement of the computer application program development process, software testing methods are becoming more and more abundant and systematic to test the accuracy, integrity, and safety of the program. The applicable scope of the digital music classroom teaching assistant system is music classroom education. Compared with other aspects, in order to pay attention to the accuracy of each function of the system, the main test method is black box test (also called function test), which is used to detect whether each function can be used normally.

As shown in Table 4, the test case diagram of the music score editing module is presented. The main functions of the module are shown in the table, and each function is designed with test cases and the test results are displayed.

*(1) Test Introduction*. Open and create new scores: These two functions belong to the score editing initialization submodule. The opening of music scores is mainly tested from the efficiency of reading music scores and the legitimacy of the opening of music scores. Therefore, some test cases with incorrect parameters and irregular operations are designed. All tests are normal and qualified, and the test results have been confirmed.

### 4.4. Demonstration Module Test of Music Composition

As shown in Table 5, the test case diagram of the music score demonstration module is presented. The main functions of the module are shown in the table, and each function is designed with test cases and the test results are displayed.

*(1) Test Introduction*. If you select the area loop to be played, the main test is whether there is a problem in an operation different from the previous one. The default condition of not selecting the area is to play the entire score, so the test result is normal. All the above tests are qualified and the test results have been confirmed.

## 5. Conclusion

At present, due to the rapid development of mobile networks, various related services have also attracted the attention of various industries, and its business volume has increased in an instant. Behind this hot phenomenon, people's requirements for cellular communication systems are also increasing. In order to meet the needs of people's lives, they are moving toward continuous expansion of capacity, continuous improvement of operation speed, and continuous acceleration of system response to changes in the line of defense. Facing people's new requirements for the network, the LTE and WiMAX standard groups were introduced based on the existing service desks to improve the operating efficiency of the system spectrum, continuously expand the system capacity, reduce the carrying capacity of the heat source station itself, and continuously increase the indoor network coverage area, thereby further improving the quality of service (QoS). This kind of network architecture composed of macro-base stations and micro-base stations is called a heterogeneous cellular network. At the same time, energy efficiency is based on global warming and operating cost management considerations and has become another important performance indicator of wireless communication systems. Based on this, this topic starts from the current situation of music classroom education in the digital and information age and analyzes many problems existing in the current music classroom education process. After comparing and analyzing the current popular music education software, this article designs an educational assistant system for music classroom education and selects the most suitable computer technology to implement it according to the characteristics of the system itself. The system integrates the StarC cloud platform of a certain school, which is suitable for music education in many schools and has achieved good results.

After establishing the audio data deployment strategy, simulation method, and architecture design based on heterogeneous cellular network, this paper designs the corresponding music composition teaching system, mainly including score editing, viewing, and content display of the composition teaching system, and the final test shows that the system designed in this paper can be effectively used in various music school teaching forms combined with heterogeneous cellular networks.

## Figures and Tables

**Figure 1:** Using 7-dimensional features to train a random forest.

**Figure 2:** Using 1572-dimensional features to train a random forest.

**Table 1:** Characteristics of various types of base stations in the LTE-A heterogeneous cellular network.

Base station type	Deployer	Transmit power configuration	Coverage radius	Return trip	Scene use
Picocell	Operator	23∼30 dBm	<300 m	X2 interface	Hot spot coverage
RemoteRadioHead	Operator	46 dBm	1∼25 km	Optical fiber	Basic coverage

**Table 2:** Comparison of the test results of the two classification systems using the TUT data set.

Features and decision models	Flat measurement index			
	Ambient sound accuracy (%)	Environmental sound recall rate (%)	Music accuracy (%)	Music recall rate (%)
7-dimensional features + 3sigma judgment	76.19	38.01	72.22	93.14
1572-dimensional features + decision tree decision	84.60	96.07	97.54	89.90

**Table 3:** Comparison of the test results of the original classification system, decision tree model, and random forest model using the TUT data set.

Features and decision models	Flat measurement index			
	Ambient sound accuracy (%)	Environmental sound recall rate (%)	Music accuracy (%)	Music recall rate (%)
7-dimensional features + 3sigma judgment	76.19	38.01	72.22	93.14
1572-dimensional features + decision tree decision	84.60	96.07	97.54	89.90
46-dimensional features and random forest model after feature selection	94.61	94.06	96.58	96.90

**Table 4:** Test case list of music score editing module.

Function description	Use case description	Test results	Test result
Open sheet music	(1) Open various types of music scores	(1) Various types of music can be opened normally to ensure the reading speed of music	Qualified
	(2) Open another score while editing the score	(2) If you open another score during the editing process, you will be asked to save the currently edited score first	
	(3) Prepare to open the file in other forms	(3) The system is set to only support specific types of music opening	
	(4) Open the score of this article	(4) Open the empty worksheet to show that the worksheet is empty	

New score	(1) When inputting music score information, add special characters or set very long or very short (2) Please try to set the playback speed and the number of audio tracks to infinitely high or infinitely small	(1) Prompt “Is the input format available, please re-enter” (2) The playback speed and the number of audio tracks can only be set within a certain range (3) All the previously set information has been saved (4) The editing module must be updated to the state before the build	Qualified
	(3) After setting the staff information, return to the music information to confirm whether the previous settings are saved		
	(4) Cancel the creation of new music before completion		

Add notes and dots	(1) Try various combinations of notes (2) Try various combinations of notes and dots (3) Add additional points separately	(1) Prompt “Music score is Ning” (2) Prompt “You can add notes or points to the current position” (3) The combination method does not comply with the rules of music Prompt “Cannot add notes” (4) If the combination of dots and notebooks does not meet the music rules, it will prompt “Cannot add dots.”	Qualified


Drag and drop to modify the clef, key signature, and time signature	(1) Drag and drop to change the order of note symbols, pitch, and beat (2) Drag the musical part symbols, keys, and beat symbols to other notes (3) Different beat numbers of different music tracks with more than 1000 music tracks (the original requirements are the same)	(1) All changes are normal	Qualified
		(2) Drag to other places will display a warning	
		(3) Drag onto the audio track; other audio tracks will change accordingly	

Save the score	(1) No editing guarantee after creating a new score (2) Change the file extension when saving (3) After the score is saved normally, open the score again (4) After the [Save] dialog box is displayed, click [Cancel]	(1) Prompt “Music score is empty”	Qualified
		(2) Prompt “The suffix name does not meet the rules”	
		(3) The music can be displayed normally	
		(4) The music enters the state before saving	

Preview the score	(1) Scale the score in different proportions	(1) The score changes normally according to the scale of enlargement and reduction	Qualified
	(2) Adjust the playback sound and speed during music playback	(2) The reproduction effect will change according to the adjustment of the reproduction speed and sound	

**Table 5:** List of examples for viewing and trial of the score demo module.

Function description	Use case description	Test results	Test result
Select the track, pitch, and instrument of the score to be played	(1) Select an audio track, or not select an audio track, or select a specific audio track to display rendering	(1) After selecting the audio track to be used, all audio tracks will be displayed on the score. If no track is selected, the score is empty	Qualified
	(2) Set different tones according to the audio track	(2) After setting different tones, the score will be displayed normally	
	(3) Set different instruments according to the audio track	(3) Set music when playing various instruments	

Loop playback of specific sections of the score	(1) Select a single area, multiple areas, all areas and zero areas for loop playback	(1) If one or more areas are selected, a single area is looped; if zero or all areas are selected, all areas are played	Qualified
	(2) After selecting several areas, cancel all areas and play	(2) Play all	

Piano display and switching	(1) Cancel the piano display after changing the position	(1) Although the piano is hidden, the music score occupies the entire interface	Qualified
	(2) After canceling the display, switch the position of the piano and the score	(2) The switch button is not active and cannot be switched	
	(3) If there is no music, please cancel the display	(3) The piano is hidden and the interface is empty	
	(4) There is no music when the position of piano and music is switched	(4) The switch button cannot be completed in the inactive state	

Scale of the score	(1) Expand the score	(1) After zooming in to a specific situation, you cannot zoom in again (2) After locked to a certain level of LJ, no further reduction is allowed (3) The operation cannot be completed when the zoom button is inactive	Qualified
	(2) Reduce the score		
	(3) Zoom in or zoom out when there is no music		

Linked music score and piano playback	(1) If the link is over, cancel the display of the piano, and then return the display of the piano to its original position.	(1) Normally cancel and resume display after normal playback (2) The reproduced sound will change when the sound is adjusted, and the speed will also change when the speed is adjusted (3) After the change, the score will be reloaded and can continue to play together (4) Except for some special musical scores, there are no problems with other musical scores. All vocalizations are normal	Qualified
	(2) Adjust the reproduction speed and sound during link reproduction		
	(3) After playing the link, zoom in and zoom out the music		
	(4) When playing the link, switch the position of the score and piano		
	(5) When playing together, change the playing track, pitch, and instrument		
	(6) Play other music and confirm whether the display and sound of the music are correct		

## Data Availability

The datasets used and/or analyzed during the current study are available from the author upon reasonable request.
